# The Effect of Flowable Composite Resins on Periodontal Health, Cytokine Levels, and Immunoglobulins

**DOI:** 10.1155/2022/6476597

**Published:** 2022-04-23

**Authors:** Cem Peskersoy, Aybeniz Oguzhan, Onder Gurlek

**Affiliations:** ^1^Ege University, Faculty of Dentistry, Department of Restorative Dentistry, Turkey; ^2^Ege University, Faculty of Dentistry, Department of Periodontology, Turkey

## Abstract

**Objective:**

This study investigated the effects of flowable resin composites (FCR) on the restoration of noncarious cervical lesions (NCCL) and their impact on periodontal tissues.

**Materials and Methods:**

30 periodontally healthy patients were assigned into three groups randomly; group VF: self-adhering FCR, group NF: fluoride-releasing FCR, and group SF: microhybrid FCR. Gingival crevicular fluid (GCF) volume levels of osteoprotegerin (OPG), immunoglobulins (IgA, IgM), and interleukins (IL-1, IL-1*β*, and IL-10) in GCF were analyzed with ELISA tests. Clinical success rates were evaluated using USPHS criteria during the 12-month follow-up.

**Results:**

The GCF volume was increased mostly in group SF (1.34 ± 0.09 *μ*l). While the titer of interleukin was increased in all groups, higher increases were observed in IL-1 and IL-1*β* in group NF (170.78 pg/ml and 39.35 pg/ml). Increased IL-10 was observed in group VF (14.33 ± 0.85 pg/ml). IgA levels varied partially among all groups (*p* > 0.05), and even IgM levels were elevated immediately after the restoration process but returned to normal on the 28th day (*p* < 0.05). Group NF failed in most of the USPHS criteria, while the material group VF and group SF presented acceptable results except in the marginal adaptation criterion (*p* < 0.05).

**Conclusions:**

Clinical efficacy of self-adhering FCR was found the best for restoration of NCCL while fluoride-releasing FCR stimulated the periodontal response and had negative effects on GCF volume, cytokine, and immunoglobulin levels.

## 1. Introduction

Flowable composite resins (FCRs) have been designed for use in instances where the geometry and conditions of a cavity are not always ideal [1]. FCRs were created while developing adhesive technology to prevent polymerization shrinkage and form a stress-breaking barrier [1, 2]. Recently, adhesive technology has begun to be integrated into the material to reduce the application steps and increase the clinical performance of flowable composites, such as abrasion and fracture resistance and bond strength [3]. As a result, “self-adhering” and low-viscosity FCRs have been introduced to the market. In addition, developers thought that these materials could have high fracture resistance and stretching capacity due to their low elasticity modulus, as well as their frequent use as force breakers under restoration in Class I and II cavities and carious and noncarious cervical lesions (NCCLs) [2, 4].

FCRs' filler content (57–78% by volume) is lower than that of conventional composites (81–92% by volume), which prevents the reduction of undesirable polymerization shrinkage in the material [5, 6]. Polymerization shrinkage impairs the adaptation of the composites to cavity walls, meaning micro- and nanogaps may occur [6]. These gaps bring major problems in terms of both adhesion and bacterial colonization, which leads to postoperative sensitivity, microleakage, plaque accumulation, secondary caries formation, and restoration failure [6]. To overcome these problems, manufacturers have added antibacterial properties to resin composites and adhesive systems [7]. The most frequently applied improvement in resin composites is giving the material an ion-releasing structure [3]. Although this application yields positive results in the short term, knowledge of its effect on the success of the material remains limited in the long term [3].

Despite the recent development of technologies and options in the FCR field, the most important issues still under investigation are biocompatibility and antimicrobial efficacy. Resin composite materials, especially for use in Class V cavities, come in direct or indirect contact with various tissues, such as pulp, gingiva, tongue, and buccal mucosa. Therefore, for these materials to be used safely in the mouth, they should not have cytotoxic, mutagenic, or carcinogenic effects or trigger an inflammatory response from host cytokine and immunoglobulin release mechanisms [8].

Cytokines are low molecular weight proteins synthesized in response to biological, chemical, or physical factors that induce and maintain a localized inflammatory response [9]. IL-1 and IL-1*β* are two of the main proinflammatory (inflammation-triggering) cytokines that are triggered even after probing and scaling processes and thus have a dominant role in periodontal destruction [10]. In addition, IL-1 induces its own release from macrophages and thus plays a role in increasing immunoglobulin levels [10]. IL-10, meanwhile, suppresses the uncontrolled destruction in tissues and the biological activities of proinflammatory cytokines. This single mechanism within the immune system to suppress IL-1 activity ensures that inflammation is kept under control [9, 10]. However, these mediators in gingival crevicular fluid (GCF) and saliva have a very short half-life, as well as a high rate of increase. IL-1 is one of the cytokines with the longest half-life at 15 hours, while it is 2.5 hours for 1L-1*β* and 2–5 hours for IL-10 [9]. Immunoglobulins' half-lives are longer, taking 5–8 days for IgM and 6–11 days for IgA [9]. For this reason, in examining cytokine levels in oral tissues, more short-term studies have been conducted since mediator levels reset in the long term [11].

Clinical trials are important tests to evaluate the clinical efficacy and biocompatibility of restorative materials. Therefore, this study is aimed at evaluating the clinical success of cavity restoration using three different properties of FCRs and their biological effects on the surrounding tissues in Class V caries-free cervical region root surface lesions. The materials tested in this study are self-adhering and fluoride-releasing resin composites compared to conventional microhybrid FCRs. The study's hypothesis is that each tested material will increase cytokine and immunoglobulin levels in GCF compared to the initial level at the end of the restoration and during the follow-up period.

There are a few studies in the literature that examine the effects of resin composites on gingival and periodontal tissues and investigate mediators in [8, 12–14]. However, these studies generally focus on the levels of some cytokines, which are indicators of attachment loss and inflammation in GCF; immunoglobulin (IgM, IgA, and IgG) levels are not examined in detail. No report has been published that examines the effects of FCRs on inflammation-initiating (IL-1, IL-1*β*) and suppressing cytokines (IL-10), immunoglobulins (IgA, IgM), and osteoprotegerin (OPG) as an osteoclastic inhibitor.

## 2. Materials and Methods

### 2.1. Patient Selection

A pool of 50 randomly selected patients, aged 25–50, with Class V NCCLs was prepared. All patients were informed about the study, and written consent forms were obtained prior to the study according to ethical committee approval (No.: 29.10.2020/2020.5.1). Thirty random patients suffering from at least 4 dental NCCLs in the incisors and premolars were selected for participation. The patient inclusion criteria were as follows: (1) no restorations with related teeth; (2) no systemic disease and not under medication; (3) no symptoms of hypersensitivity or pain; (4) no signs of pulpitis or root canal treatment; (5) no bleeding during probing processes (i.e., while receiving periodontal treatment); and (6) normal occlusion (natural antagonist teeth). The NCCLs' positions were similar for each case, within a supragingival margin of 0~1 mm and featuring a defect deep into the middle layer of the dentin. Individuals with chronic diseases, who were pregnant, smoked, and/or had periodontal disease (gingivitis or periodontitis), were excluded from the study.

### 2.2. Restoration Procedure

The teeth with NCCLs for each patient were divided into three groups according to the type of FCR material to be used; 30 restorations in each group for a total of 90 restorations were made (Table 1). Three teeth of each patient with similar lesion dimensions and proximity to the gingival margin were selected for restoration. The cavities were prepared with a high-speed handpiece using diamond burs under constant water cooling at an angle of 45° at the enamel level and beveled at a width not exceeding 2 mm. Selective etching with 35% orthophosphoric acid (Scotchbond Etch, 3M Espe, MN, USA) for 30 seconds and a single-step universal adhesive system (Single Bond Universal, 3M Espe, MN, USA) were applied to the cavities prior to the FCR selection (Figure 1). For composited restoration, the prepared teeth were insulated with rolled cotton pads and polymerized using a 1200 W light source (Elipar, 3 M- ESPE, MN, USA) for 20 seconds. Then, each tooth was randomly assigned to a different group for restoration with at least two layers of composite using the appropriate FCR material. Finishing and polishing were completed using diamond finishing burs and polishing discs (Sof-Lex, 3M-ESPE, MN, USA). At the end of the restorations, the clinical findings and evaluations from the first-week, first-month, and first-year postprocedure were assessed according to the criteria of the United States Public Health Service (USPHS; Table 2).

### 2.3. Specimen Collection

GCF samples were taken from the patients within the scope of the study to determine the volume of the restored tooth before the restoration procedures, immediately after the restoration, and on days 7 and 28 posttreatment (Figure 2). The GCF samples were taken with standard-size paper strips (Periopaper, OraFlow Inc., NY, USA) after isolating the periphery of the identified teeth with rolled cotton pads to prevent saliva contamination. The paper strips were placed in the sulcus no more than 1 mm and left for 30 seconds until the patient felt moderate pressure. Strips contaminated with blood were not included in the study. The obtained paper strips were placed in Eppendorf tubes containing 1000 *μ*l saline with the help of an automatic pipette (Pipette, Borox, BeyanLab, Istanbul, Turkey) and kept at -20°C until biochemical analysis. A total of 84 GCF samples were taken from each patient, 4 for each of the three treated teeth and 1 different sample for each test parameter.

A Periotron 8000 (Oraflow, NY, USA) device was used to determine GCF volume. Before each paper strip was read, the device's calibration was checked, and the conductors were wiped with alcohol to prevent possible erroneous readings. The obtained Periotron data were converted to microliters (*μ*l) using the “MLCONVRT” software previously loaded on the computer.

### 2.4. Biochemical Analyses (ELISA Tests)

Proinflammatory mediators IL-1, IL-1*β*, anti-inflammatory mediator IL-10, immunoglobulin IgA and IgM, and mediator OPG levels that suppress osteoclastic activity in the GCF samples stored at -20°C were examined with the help of ready-made kits. For this purpose, samples stored at -20°C were left at +4°C to thaw 24 hours before the working day. For the separation of GCF from the Periopapers, the samples were vortexed for 1 minute (Vortex, Velp Scientifica, Italy) and centrifuged at 3000 rpm for 10 minutes (SK962, SinoThinker, Shenzhen, China) prior to analysis. For the determination of IL-1, IL-1*β*, IL-10, IgA, IgM, and OPG levels, ELISA kits specific to each mediator (Sunred Biotech. Co, Shanghai, China) were used according to the manufacturer's instructions. Microdilution plates were previously coated with antibodies specific to each mediator. Predetermined test steps were performed in accordance with the manufacturer's instructions with commercial kits operating on the basis of the Streptavidin-HRP double antibody sandwich technique.

### 2.5. Clinical Examination of Restorations

The clinical conditions of all restorations were followed for 12 months and evaluated according to USPHS standards. The major criteria for a successful restoration were as follows: surface gloss and roughness; surface and marginal coloration; color compatibility; integrity of anatomical form; retention of restoration; marginal adaptation; and secondary caries formation. Hypersensitivity to hot and cold stimuli, spontaneous pain, and pulp vitality were also recorded. The treatment was considered a failure if any of the major criteria presented a Charlie (bad) score.

### 2.6. Statistical Analyses

The data obtained in the study were analyzed with the SPSS 24.0 (IBM, Chicago, IL, USA) software. The conformity of biochemical and clinical variables to normal distribution was analyzed by the Kolmogorov-Smirnoff test (*n* = 20). Statistical analyses were performed using nonparametric tests, since most of the parameters examined did not show normal distribution. The differences between the groups were determined with the Mann–Whitney *U* test, and the differences between the measurements based on time were determined with the Wilcoxon signed-rank test. Correlations between clinical and biochemical parameters were analyzed by Spearman's rank correlation analysis (*p* < 0.05).

## 3. Results

In our study, 90 restorations made with three different FCR's with a total of 30 participants (11 men and 19 women) were examined. Changes in biochemical parameters obtained from GCF before and after treatment, as well as on the 7th and 28th days, are given in Table 3. The clinical evaluations at the 7th day, 28th day, 1st month, and 12th month follow-up periods after the restorations are given in Table 4.

### 3.1. Results of Biochemical Parameters

Due to Spearman's rank correlation, a significant positive correlation was seen between IL-1 levels, marginal adaptation, and discoloration (*p* < 0.05). Also, the correlation between Il-1*β* and surface roughness of the restorations was found statistically significant (*p* < 0.05). Among the markers, positive correlations between pretreatment and 1-month follow-up were observed in levels of GCF volume, IL-1*β*, and Il-10 (*p* < 0.05).

#### 3.1.1. Results of Gingival Crevicular Fluid (GCF) Volumes

The mean initial GCF fluid volume before the restorative treatment in all groups was determined as 0.97 ± 0.092 *μ*l (Table 3). After the restorations were completed, there was a significant increase in GCF volume in all groups (*p* < 0.05). The highest GCF volume was reached at the end of the 1st week in group NF (1.58 ± 0.09 *μ*l), while the GCF volumes were equalized to the baseline by the 28th day in all groups (*p* > 0.05).

#### 3.1.2. Results of Interleukin (IL-1, IL-1*β*, and IL-10) Levels

Initial interleukin levels, IL − 1 = 32.23 ± 11.40 pg/ml, IL − 1*β* = 7.81 ± 3.49 pg/ml, and IL − 10 = 5.02 ± 1.73 pg/ml, were increased in all groups (400% in IL-1, 500% in IL-1*β*, AND 300% in IL-10), after the restoration procedures (*p* < 0.05) (Table 3). However, the difference in increased IL-1 levels between the groups was not statistically significant after the operation phase (*p* > 0.05). On the 7th day, a significant decrease began in IL-1 levels, and the differences between all groups became significant on the 28th day (*p* < 0.05). The highest level of IL-1 was reached on day 7 (170.21 ± 11.60 pg/ml) after treatment in group NF, while it has not reached the initial values even at the end of the 28th day (*p* < 0.05).

The IL-1*β* level reached the highest value (39.44 ± 6.31 pg/ml) in group NF, after treatment, while the values on the 7th and 28th days (31.05 pg/ml and 16.13 pg/ml) were significantly different and higher than the other groups (*p* < 0.05). While there was a significant increase in IL-10 levels in all groups after treatment (*p* < 0.05), a significant decrease was observed in IL-10 levels as of the 7th day. Considering the IL-10 levels on the 28th day after treatment, no significant difference was found between the groups (*p* > 0.05).

#### 3.1.3. Results of Immunoglobulin (IgA and IgM) Levels

IgA and IgM levels in GCF were compared with the Mann–Whitney *U* test between groups, and with the Wilcoxon signed-rank test for time-dependent within-group changes. Mean baseline IgA (2.55 ± 0.82 mg/ml) and IgM (0.94 ± 0.41 mg/ml) levels were determined for all groups (Table 3). While there was a significant increase in IgM values after the restorations in all groups (*p* < 0.05), the increase in IgA levels and the decrease between the 7th and 28th days were not statistically significant (*p* > 0.05).

When IgA levels are examined, the highest value was observed in the group VF on the 7th day (2.72 ± 0.38 mg/ml) after the restoration procedure (*p* > 0.05); however it has reached the initial values at the end of the 28th day in all groups (*p* > 0.05). As for the IgM values, the highest values (1.35 ± 0.29 mg/ml and 1.23 ± 0.20 mg/ml) were reached after treatment in group VF and group NF (*p* < 0.05). Only in group NF, there was an increase in some cases (*n* = 7) on the 28th day, but it was not found to be statistically significant (*p* > 0.05) (Table 3).

#### 3.1.4. Results of Osteoprotegerin (OPG) Levels

The mean initial OPG levels were determined as 72.10 ± 14.46 pg/ml (Table 3). OPG values increased in all groups following the restoration and reached their highest values at the end of the 28th day (*p* > 0.05), when the intragroup values of OPG levels are examined; while a significant difference was found between all groups after treatment (*p* < 0.05), the differences between the groups at the same measurement times were not significant (*p* > 0.05). The highest OPG level was reached in group SF on the 28th day (184.66 ± 11.48 pg/ml) after treatment.

### 3.2. Results of Clinical Evaluations

Clinical examinations were performed post-op (day 1), at the 1st and 12th months according to the modified USPHS criteria (Table 4). After 12 months, only 10 of the 90 restorations (VF: 3 cases, NF: 5 cases, and SF: 2 cases) had to be replaced due to unacceptable clinical parameters.

#### 3.2.1. Surface Gloss and Roughness

According to USPHS criteria in terms of surface gloss and roughness, 26 restorations out of 30 in group VF scored as Alpha (*excellent*) after month 12 (86.7%). Three restorations (10%) in group NF and only one restoration (3.3%) in group SF have failed/scored as 3-Charlie (*unacceptable*) after 12 months.

#### 3.2.2. Marginal Coloration

In group VF, while 29 restorations (96.7%) scored 1-Alpha (*excellent*) at week 1, after 12 months, 5 restorations scored 2-Beta (*acceptable*), and 3 restorations failed 3-Charlie (*unacceptable*) with a success rate of 73.3 (*p* < 0.05). Similar to these results, in group NF only 20 restorations (66.7%) scored 1-Alpha (*excellent*), and 6 restorations (20%) scored 2-Beta (*acceptable*) at the end of the trial (*p* < 0.05). The failure rate of restorations in group SF is relatively lesser than that in all groups (1 out of 30, 3.3%).

#### 3.2.3. Color/Shade Matching

In group SF, only 1 restoration (3.3%) failed in the color/shade matching criterion at the end of 12 months (*p* < 0.05). In addition, 7 restorations (23.3%) in group NF scored 2-Bravo (*acceptable*), which was statistically significant when compared with the scores of all groups (*p* < 0.05). The 1-Alpha (*excellent*) scores presented no significant differences at different intervals (*p* > 0.05). In the 12th month, 16 restorations (17.7%) were repolished, and 8 restorations (8.88%) were replaced due to failure in marginal discoloration of color/shade mismatch.

#### 3.2.4. Anatomical Form

After 12 months, 75 restorations (83.3%) in all groups scored 1-Alpha (*excellent*) while 15 restorations (16.7%) scored 2-Bravo (*acceptable*). Anatomical form is one of the two basic USPHS criteria for secondary caries, for which the differences between and within the groups are not statistically significant (*p* > 0.05).

#### 3.2.5. Retention of Restorative Material

The survival rate of the restorations in group VF was 100.0% after 12 months, while 2 restorations (6.6%) in group NF and 1 restoration (3.3%) in group SF failed to survive (*p* < 0.05). Besides, the differences in 2-Bravo (*acceptable)* and 3-Charlie (*unacceptable*) scores between group VF and the other two groups were found statistically significant (*p* < 0.05).

#### 3.2.6. Marginal Adaptation

Marginal adaptation was the criterion with the highest number of failures among all evaluation USPHS criteria. While marginal adaptation and coloration results were found to be compatible with each other for group VF and group NF, there was no similarity for group SF (*p* > 0.05). The only restoration that needed to be replaced at 6 months due to the failure in the marginal adaptation criterion was in group NF. However, the 1-Alpha (*acceptable)* scores of group SF (27 out of 30) were found statistically different among all groups (*p* < 0.05). After 12 months, 5 restorations in group NF (5.6%) scored 3-Charlie, and the differences between the other two groups were found significant (*p* < 0.05).

#### 3.2.7. Secondary Caries

Although, after 12 months, no secondary caries formation was observed, partial demineralization (white spot lesion) was observed in 1 case in group VF and in “2” cases in the other groups, which was statistically insignificant (*p* > 0.05).

## 4. Discussion

Recent studies have reported that resin composites are a suitable alternative to adequate restoration in the treatment of NCCLs [1, 4]. Since there are no caries or bacteriological factors in these cases, the most important factors for NCCLs are adhesion, sealing, and biocompatibility [15, 16]. Consistent with the minimally invasive treatment approach, the use of resin composites in the treatment of NCCLs allows for more conservative restorations [17]. In addition, it has been shown that the resistance to abfraction forces increases when more flexible and less viscous FCRs are used in the restoration of stress-bearing posterior region teeth [18]. However, FCRs have some major shortcomings due to their lower filler content than conventional resin composites.

This study is aimed at evaluating the effects of FCRs on cytokine, immunoglobulin, and OPG levels in GCF and their clinical success when used for Class V cavities. In light of the data obtained from this study, all composite resin materials used cause an increase in IL-1, IL-1*β*, IL-10, and OPG levels in GCF. However, only a partial increase was observed in IgA and IgM levels. Since it is known that adhesive systems containing Hema promote IgG synthesis, IgA and IgM are the main immunoglobulins examined in this study [19]. Clinically, all restorative materials showed good and acceptable results according to USPHS criteria after 12 months of follow-up; of the 90 restorations, 17 were repaired, and 9 were replaced.

The polymerization process is the main sore point of resin-based composites (RBCs) [20]. Many factors affect this process, from the type of filler and methacrylates in the RBCs to their volume, from the application technique of the restoration to the application area, and from the viscosity of the material to the curing process [6, 20]. As a result of insufficient polymerization, negative consequences such as shrinkage and microleakage may occur [20]. Polymerization shrinkage can cause gaps at the tooth restoration interfaces, which leads to bacterial invasion and secondary caries formation [6]. Inadequate curing is one of the main causes of residual monomers, especially in the cavity floor and gingival margins where light does not reach [6, 21]. Besides their low filler ratio, FCRs also increase the volume of residual monomers [21]. In FCRs whose filler ratio and viscosity are reduced for ease of application, adaptation, and fluidity increase, the mechanical properties of the material and its biocompatibility to gingival tissues also decrease [22].

RBCs with antibacterial effects have been developed to manage plaque accumulation and secondary caries caused by polymerization shrinkage [7]. Additionally, it is thought that they favor the remineralization process through fluoride ion release and induce the antimicrobial mechanisms of the host [7]. However, ion-releasing RBCs, which have been introduced as an alternative restorative material for these purposes, do not achieve the desired success in Class V cavities in every case [23]. Studies have shown that the release of fluoride ions provides antibacterial activity only for a certain period of time [24, 25]. In a study by Kwon et al. of resin-based luting cements and in another study by Kanjevac et al. of glass ionomer materials, the researchers showed that fluoride ions cause a reaction in both pulpal and periodontal cells and trigger the release of inflammatory cytokines, especially IL-1 and IL-1*β* [12, 26]. The current study examined the effects of fluoride-releasing restorative materials on interleukins (IL-1, IL-1*β*, and IL-10) and immunoglobulin levels. Although rapid increases in all interleukin levels for all FCRs were observed, interleukin levels in the fluoride-releasing FCR decreased after 1 month but were still higher than that in the other groups. The most likely explanation for this situation is that the material continues to release fluoride for at least 1 month, and this led to a continued inflammatory response.

An increase in IL-1 levels also triggers the release of the anti-inflammatory cytokine IL-10 to restrain the increase of inflammation and tissue destruction [27]. Kamalak et al. showed that after 24 hours of applying two different FCRs, the IL-6 and IL-8 levels secreted from the cells were balanced by increased IL-10 secretion [28]. Similarly, in this study, a significant IL-10 storm was detected in all groups at the end of the first day and increased up to 3-4 times from the baseline. This could be explained by the remaining unpolymerized methacrylate monomers in the contents of the FCRs triggering a foreign body response (FBR) in the host and thus causing increased cytokine levels. This increase also stimulated IL-10 release, which was supposed to slow the inflammatory process. However, the chemical properties of the FCRs led to continued inflammation for 1–4 weeks. In addition, clinical studies show that IL-1beta promotes inflammatory response and destruction of the alveolar bone by increasing osteoclast formation [29]. Higher IL-1*β* levels of GCF are seen as a sign of periodontal disease, and studies proved that periodontal tissue breakdown may be controlled by regulating IL-1*β* expression. In our study, IL-1*β* levels were found to be higher than the baseline at the end of the observation period in the NF group. This may be due to the fact that the fluoride release activity of the material lasted longer than expected and possibly promoted IL-1*β* release. Therefore, in the restoration of deep subgingival cavities with FCRs, it is necessary to be selective in the use of resin-containing materials, as they will increase the expression of Il-1*β*.

The second major problem that RBCs have to overcome is bonding (adhesion) to dental hard tissues. For this reason, self-adhering flowable composites have been introduced to increase the bonding and adhesion of FCRs by adding acidic functional monomers such as glycerol phosphate dimethacrylate (GPDM) or 4-methacryloyloxyethyl trimellitic acid (4-META) [30]. Anderson et al. stated that methacrylates in the adhesive systems used for the adhesion of RBCs increase interleukin levels due to their toxic properties while increasing some immunoglobulin levels [19]. Other studies examining the effects of different monomers, such as TEGDMA and UDMA on human cells, have determined that they cause high cytokine release [31, 32]. However, there are studies showing that 4-META and GPDM monomers can be used safely on pulp tissue without triggering a cellular inflammatory response [33]. The findings of this study also support these results, that possibly UDMA-containing, self-adhering FCR stimulates IL-1 and IL-1*β* secretion similar to that of ion-releasing restorations. In addition, only in the self-adhering FCR did a partial increase in IgM levels occur after the restoration phase. This may be a result of GPDM monomers in self-adhering FCRs triggering a localized IgM response and causing their rapid increase. IgM antibodies seem to have a high tendency to bind to glycosylated molecules, showing that the glycerophosphate backbone of the GPDM monomer is a prime target [34].

OPG, which plays an active role in the mechanism of bone destruction resulting from periodontal disease, also suppresses osteoclastic activity [35]. OPG generally increases in cases where the osteoclastic-osteoblastic cycle is intensely observed, such as during periodontal treatment, surgical procedures, and orthodontic applications [35]. The number of studies examining the effects of resin composites on OPG is negligible [11, 35]. Initially, the increased OPG levels observed in the current study were considered a consequence of the body's anti-inflammatory response to periodontal tissue trauma during the restoration process and would decrease over time. Despite this, the continued increase in OPG levels during the 1-month follow-up period raised the idea that the damage to the periodontal and bone tissues may be permanent during the finishing of the restorations. However, some studies have demonstrated an increase in OPG levels after certain dental treatments, which might indicate the possible involvement of OPG in the regulation of periodontal tissue repair that could last up to 6 months [11, 36]. Similar to the increase in OPG, this study also revealed a significant increase in GCF after the restoration procedures. There are multiple possible explanations for changes in GCF volume, such as periodontal scaling, surgical procedures, and restorative treatments [1, 13]. Celik et al. reported that resin composite, compomer, and glass ionomer cements applied to Class V cavities caused increased GCF volume that continued to rise during the study's 3-week follow-up period and claimed that this may be due to the chemical content of the restoration materials [8]. In the current study, the highest increase was observed in the fluoride-releasing FCR, but a significant increase in GCF volume was detected in all FCRs. A normalization in GCF volume also occurred, with the fluoride-releasing capacity of the FCRs decreasing over time, in which Tuncer's studies also supported this argument [37].

Studies examining the effect of resin composites on oral immunoglobulins are very limited [38, 39]. In those that do exist, partial increases were found in immunoglobulin G (IgG) and secretory immunoglobulin A (s-IgA) levels [40]. Similar results arose in this study, and a partial increase in immunoglobulin A and M (IgA, IgM) levels did occur. The most likely reason for the lack of significant changes in immunoglobulin levels is that the patient had periodontal treatment before the operative procedure. In individuals with periodontal disease, an increase in acute immunoglobulin levels has been observed after traumatized dental treatments, such as scaling, deburring, subgingival curettage, and restorative treatments [38–40].

When RBCs are used in teeth that carry heavy chewing loads and occlusal stresses in the posterior region, there are many factors that affect their clinical success [3, 5, 6, 16]. In this randomized clinical study, the factors affecting the clinical success of different types of FCRs used to treat NCCLs were evaluated per USPHS (Ryge) criteria. The low filler ratio of FCRs causes a decrease in their viscosity, as well as a decrease in mechanical properties, such as marginal maladaptation and deformation on surface roughness [2]. Especially as a result of the decreased compression, tensile, and wear resistance, cracks, fractures, and failures can be seen in FCRs performed in NCCLs over time [18]. Similarly, in this study, there were significant decreases in surface smoothness, marginal adaptation, and marginal coloration criteria at the end of the twelfth month in all groups. This can be attributed to FCRs alone not being able to sufficiently resist heavy occlusal loads and ongoing abrasive factors. Extant studies have shown that more successful clinical results are possible when flowable composites are used together with nanohybrid conventional composites [5]. Additionally, it has been determined that fluoride-releasing composites were more deformed and had rougher surfaces at the end of a 12-month period compared to the other groups. These findings are compatible with the results of Kavaoglu's study in which the chemical structure of the fluoride-releasing RBC deteriorated over time and the material's resistance to abrasion and wear decreased [41]..

The main negative effects of FCRs' low filler ratio are increased polymerization shrinkage and higher water absorption [6, 16]. The increase in polymerization shrinkage negatively affects both aesthetic and hygienic parameters, such as marginal adaptation and coloring. In addition, higher organic matrix content increases water solubility and leads to more wear and defect formation, which affects the long-term performance of the restoration [42]. This increased solubility and decreased wear resistance also lead to the rapid coloring of the FCRs due to water absorption [16]. There are also studies showing marginal gaps and voids in FCRs as consequences of polymerization shrinkage, which traps coloring liquids more easily and causes rapid discoloration of resin composites [5, 16]. The fluoride-releasing FCR used in this study underwent more color changes during the 12-month follow-up. The changes in the chemical structure of the material over time depending on the fluoride release and relatively low filler ratio (60%) could be responsible for these failures.

Within the limitations of this study, the levels in GCF of 4 cytokines and 2 immunoglobulins, which play a role in periodontal inflammation, after the construction of flowable composite restorations were investigated. Examination of other major cytokines such as IL-6, TNF-*α*, and RANKL that directly affect inflammation in future studies will provide more comprehensive and definitive results explaining the relationship between resin composites and periodontium. Also, the guidelines of the American Dental Association (ADA) have suggested that at least 18-month long-term follow-ups are required to fully demonstrate the success of RBC materials [3]. In the current study, the failure rate was below 5% in the VF and SF groups, while it was 6.5% in the fluoride-releasing composite (NF) group. Therefore, long-term clinical follow-up is needed to fully evaluate the success of both self-adhering flowable composites and fluoride-releasing resin composites.

## 5. Conclusions

The low viscosity of FCRs' permits ease of use, while it can easily overflow into periodontal tissues and cause localized inflammation. Methacrylate, silica-based fillers, and the ion-releasing organic matrix in the contents of RBCs increase interleukin levels in the surrounding periodontal tissues and GCF after polymerization. The use of self-adhering composites together with an additional adhesive system increases the probability of residual monomers, thus causing IL-1 levels to increase more if conventional composites had been used. The antibacterial effect of fluoride ion-releasing composites lasts for a short time, and their structural integrity weakens afterward, causing decreased marginal compliance and increased surface roughness. The low filler ratio of FCRs' diminishes its mechanical properties such as a decrease in compression, stretching, and abrasion resistance and causes cracks, fractures, abrasions, and losses over time.

## Figures and Tables

**Figure 1:** Materials used in the study. (a) Vertise flow (self-adhering FCR). (b) Nova Compo SF (microhybrid FCR). (c) Nexcomp flow (fluoride-releasing FCR). (d) Single Bond Universal (all-in-one self-etch adhesive).

**Figure 2:** Case design of the study. (a) Clinical condition of the teeth and collecting GCF before treatment. (b) Post-op. GCF sampling immediately after the restoration phase. (c) 1-week follow-up GCF collecting. (d) 1-month follow-up control and sample collecting.

**Table 1:** Materials used in the study.

Material	Brand	Group	Batch No.	Contents
Self-adhering flowable composite group 1, Vertise flow	Kerr Corp, (Orange Co. CA, USA)	VF	5079369	GPDM, 4-META, UDMA, BisGMA, photoinitiator, 70% ytterbium fluoride, barium aluminosilicate glass, colloidal silica, and prepolymerized filler
Fluoride-releasing flowable composite group 2, Nexcomp flow	Meta BioMED, (Chungbuk, S. Korea)	NF	1107222	Bis-GMA, UDMA, Bis-EMA TMPTMA, 60%, 0.8 *μ*m barium aluminum borosilicate, alumino-fluoro-silicate, and calcium-hydroxy-phosphate
Microhybrid flowable composite group 3, Nova Compo SF	Imicryl Corp. (Konya, TURKEY)	GF	15278	31% methacrylate (UDMA, Bis-MEPP, TEGDMA), 69% silicon dioxide, 50% strontium glass, pigments, and photoinitiators
Universal bonding (adhesive) system, Single Bond Universal	3M ESPE (St. Paul, MN, USA)	—	622643	MDP, phosphate monomer, HEMA, dimethacrylate resin, silane, ethanol, copolymer (polyalcenoic acid), water, and initiators
Acid (etch) gel scotch bond gel	3M ESPE (St. Paul, MN, USA)	—	3741904	37% orthophosphoric acid, benzalconium chloride

**Table 2:** USPHS (Ryge) clinical evaluation criteria.

Category	Score	Clinical evaluation criteria
Surface roughness and gloss	1-Alpha	Surface of restoration is neat and smooth
	2-Bravo	Slightly uneven and rough surface
	3-Charlie	There are deep notches and irregular grooves on the surface

Marginal coloration	1-Alpha	There is no color difference between the restoration and the tooth
	2-Bravo	There is a slight discoloration
	3-Charlie	The discoloration progresses towards the cavity

Color/shade matching	1-Alpha	No change in color, shade, or transparency of the restoration
	2-Bravo	Slight change of color (up to 2 shades)
	3-Charlie	Significant change of color (more than to 2 shades)

Anatomical form	1-Alpha	Restoration is sound and continuous
	2-Bravo	Slight discontinuity on marginal ridges but clinically acceptable
	3-Charlie	Wear and deformation in restoration are present

Retention of restoration	1-Alpha	Restoration is sound and present
	2-Bravo	Restoration has repairable cracks and/or wear
	3-Charlie	Significant parts or all of the restoration have been lost

Marginal adaptation	1-Alpha	No visible crevice and the explorer do not catch at interfaces
	2-Bravo	There is a small crevice, and the explorer falls into it
	3-Charlie	Explorer is advancing towards dentin or base of restoration

Secondary caries	1-Alpha	The tooth is sound
	2-Bravo	Localized demineralization areas are present
	3-Charlie	Secondary caries are present

**Table 3:** Gingival crevicular fluid (GCF) volumes, interleukin (IL-1, IL-1*β*, and IL-10), immunoglobulin (IgA, IgM), and cytokine (osteoprotegerin (OPG)) levels before and after treatment obtained from the study levels at 1-week and 1-month follow-ups.

Biochemical parameter	Flowable composite materials											
	Vertise flow (VF)				Nexcomp flow (NF)				Nova Compo SF (SF)			
Evaluation periods	Pre-T.	Post-T.	1 week	1 month	Pre-T.	Post-T.	1 week	1 month	Pre-T.	Post-T.	1 week	1 month
Gingival crevicular fluid (GCF) volume (pg/ml)	0.95 (0.02)	1.20 (0.07)	1.38 (0.06)^a^	*1.08* (*0.06*)	0.98 (0.03)	1.30 (0.07)	1.21 (0.15)^a^	*1.09* (*0.08*)	0.98 (0.07)	1.18 (0.07)	1.34 (0.09)	*1.12* (*0.12*)
Interleukin-1 (IL-1) (pg/ml)	31.58 (5.66)	129.84 (11.16)	115.88^b^ (11.59)	57.49^c^ (7.72)	32.28 (6.84)	137.27 (11.01)	170.21^b^ (11.60)	82.79^c^ (8.72)	33.47 (4.68)	119.68 (9.98)	92.39^b^ (8.27)	36.32^c^ (8.32)

Interleukin-1beta (IL-1*β*) (pg/ml)	7.83 (1.75)	35.97 (4.65)	17.72^d^ (4.42)	*9.23* ^e^ (*1.68*)	8.19 (1.20)	39.44 (6.31)	31.00^d^ (6.67)	*16.26* ^e^ (*1.93*)	7.41 (2.13)	36.55 (4.48)	18.23^d^ (3.22)	*8.74* ^e^ (*1.76*)
Interleukin-10 (IL-10) (pg/ml)	4.76 (0.82)	14.45 (0.84)	5.79 (0.29)	*5.50* (*0.21*)	5.16 (0.81)	12.85 (0.62)	6.04 (0.94)	*5.84* (*0.67*)	5.15 (0.94)	14.15 (0.65)	5.50 (0.10)	*5.18* (*0.14*)
Immunoglobulin A (IgA) (mg/ml)	2.56 (0.51)	2.68 (0.30)	2.72 (0.38)	2.58 (0.14)	2.61 (0.42)	2.70 (0.22)	2.59 (0.20)	2.45 (0.20)	2.48 (0.28)	2.65 (0.25)	2.56 (0.33)	2.44 (0.15)
Immunoglobulin M (IgM) (mg/ml)	0.93 (0.22)	1.35 (0.29)	0.94 (0.51)	0.92 (0.05)	0.92 (0.18)	1.23 (0.20)	0.94 (0.26)	1.00 (0.20)	0.98 (0.21)	1.13 (0.29)	1.02 (0.28)	0.96 (0.22)

Osteoprotegerin (OPG) (pg/ml)	71.68 (6.22)	108.18 (10.92)	140.55^f^ (9.65)	179.99 ^g^ (18.86)	75.48 (8.19)	112.41 (7.94)	134.90^f^ (13.14)	166.50^g^ (15.96)	69.14 (5.81)	109.51 (11.84)	153.55^f^ (19.42)	184.66^g^ (11.48)

Standard deviations are given in parentheses. Different superscript letters indicate statistical differences between groups (*p* < 0.05). Values written in italics indicate positive correlations before and after treatment.

**Table 4:** USPHS scores of restorations made with different flowable composites applied in the study after treatment (Post-op.), 1-week, 1-month, and 12-month follow-ups.

USPHS criteria	Flowable composite materials											
	Vertise flow (VF)				Nexcomp flow (NF)				Nova Compo SF (SF)			
Evaluation periods	Post-op.	1st week	1st month	12th month	Post-op.	1st week	1st month	12th month	Post-op.	1st week	1st month	12th month
Surface roughness and gloss	*1* (*A* = 30)	*1* (*A* = 28) (*B* = 2)	*1* (*A* = 27) (*B* = 3)	*1* ^a^ (*A* = 26) (*B* = 3) (*C* = 1)	*1* (*A* = 30)	*1* (*A* = 29) (*B* = 1)	*1* (*A* = 25) (*B* = 5)	2 ^a,b^ (*A* = 23) (*B* = 4) (*C* = 3)	*1* (*A* = 30)	*1* (*A* = 28) (*B* = 2)	*1* (*A* = 26) (*B* = 4)	*1* ^b^ (*A* = 25) (*B* = 4) (*C* = 1)

Marginal coloring	*1* (*A* = 30)	*1* (*A* = 29) (*B* = 1)	*1* ^c^ (*A* = 25) (*B* = 5)	*2* (*A* = 22) (*B* = 5) (*C* = 3)	*1* (*A* = 30)	*1* (*A* = 28) (*B* = 2)	*2* ^c,d^ (*A* = 21) (*B* = 9)	*2* ^e^ (*A* = 20) (*B* = 6) (*C* = 4)	*1* (*A* = 30)	*1* (*A* = 28) (*B* = 2)	*1* ^d^ (*A* = 26) (*B* = 4)	*1* ^e^ (*A* = 24) (*B* = 5) (*C* = 1)

Color/shade matching	*1* (*A* = 30)	*1* (*A* = 30)	*1* ^f^ (*A* = 28) (*B* = 2)	*1* ^g,h^ (*A* = 27) (*B* = 3)	*1* (*A* = 30)	*1* (*A* = 27) (*B* = 3)	*1* ^f^ (*A* = 26) (*B* = 4)	*2* ^g,h^ (*A* = 23) (*B* = 7)	*1* (*A* = 30)	*1* (*A* = 29) (*B* = 1)	*1* (*A* = 27) (*B* = 3)	*1* ^h^ (*A* = 25) (*B* = 4) (*C* = 1)

Anatomical form	*1* (*A* = 30)	*1* (*A* = 30)	*1* (*A* = 28) (*B* = 2)	*1* (*A* = 26) (*B* = 4)	*1* (*A* = 30)	*1* (*A* = 29) (*B* = 1)	*1* (*A* = 26) (*B* = 4)	*1* (*A* = 24) (*B* = 6)	*1* (*A* = 30)	*1* (*A* = 29) (*B* = 1)	*1* (*A* = 27) (*B* = 3)	*1* (*A* = 25) (*B* = 5)

Retention of restoration	*1* (*A* = 30)	*1* (*A* = 29) (*B* = 1)	*1* (*A* = 27) (*B* = 3)	*1* ^i,j^ (*A* = 27) (*B* = 3)	*1* (*A* = 30)	*1* (*A* = 28) (*B* = 2)	*1* (*A* = 25) (*B* = 5)	*2* ^i^ (*A* = 22) (*B* = 6) (*C* = 2)	*1* (*A* = 30)	*1* (*A* = 27) (*B* = 3)	*1* (*A* = 26) (*B* = 4)	*1* ^j^ (*A* = 23) (*B* = 6) (*C* = 1)

Marginal adaptation	*1* (*A* = 30)	*1* (*A* = 28) (*B* = 2)	*2* ^k^ (*A* = 21) (*B* = 9)	*2* ^m^ (*A* = 21) (*B* = 6) (*C* = 3)	*1* (*A* = 30)	*1* (*A* = 26) (*B* = 4)	*2* ^l^ (*A* = 22) (*B* = 7) (*C* = 1)	*2* ^m,n^ (*A* = 22) (*B* = 4) (*C* = 4)	*1* (*A* = 30)	*1* (*A* = 28) (*B* = 2)	*1* ^k,l^ (*A* = 27) (*B* = 3)	*2* ^n^ (*A* = 21) (*B* = 7) (*C* = 2)

Secondary caries	*1* (*A* = 30)	*1* (*A* = 30)	*1* (*A* = 30)	*1* (*A* = 29) (*B* = 1)	*1* (*A* = 30)	*1* (*A* = 30)	*1* (*A* = 30)	*1* (*A* = 28) (*B* = 2)	*1* (*A* = 30)	*1* (*A* = 30)	*1* (*A* = 30)	*1* (*A* = 28) (*B* = 2)

Italicized numbers present the average USPHS score of the selected criteria. Case numbers and scores are given in parentheses. (*A*: Alpha, *B*: Bravo, and *C*: Charlie). The same superscript letters indicate statistical differences between groups (*p* < 0.05).

## Data Availability

The data used to support the findings of this study are available from the corresponding author upon request.
